# Research on the Application of Animation Design Based on Machine Learning and Dynamic Image Index

**DOI:** 10.1155/2022/2690415

**Published:** 2022-06-30

**Authors:** Yaodong Yin

**Affiliations:** Department of Fine Arts, Taiyuan Normal University, Jinzhong, China

## Abstract

With the development of computer technology, animation is more and more used because of its simple, effective, and higher performance. Machine learning has become the core of artificial intelligence at present. Intelligent learning algorithms are widely used in practical problems such as evaluation. Knowledge-based automatic animation production system faces two challenges: (1) lack of learning ability and waste of data on the website; (2) the quality of animation produced that depends on the level of system designer and the inability of system users to participate in animation production.In order to solve these two problems, an active animation learning system enables the animation system to constantly learn experience and produce the most popular animation, for the first time, for animation production system design and implementation of applied research. Image retrieval technology is a research center in the field of image application. It is widely used in many fields, such as electronic commerce. Animation design will use dynamic image and machine learning to innovate.

## 1. Introduction

Animation design is based on all-weather computer-aided animation automatic production technology, which is based on computer-aided animation technology [1]. In the whole process from receiving SMS to output animation, there is no manual process. The animation design production system consists of four basic units: information extraction, plot qualitative planning (ADL), animation quantitative calculation (CAL), and network development. After receiving SMS from animation production system, the staff will process natural language text and semantic analysis text, and conduct qualitative analysis and quantitative calculation of text [2]. Finally, animation design system faces two challenges through animation demonstration and production: (1) there may be a lack of learning ability and waste of a large amount of animation short message accumulated data; (2) the quality of the animation produced depends on the design level of the system, originally designed for the animation production system, and a dynamic animation learning system has been established to enable the animation production system to continuously learn experience and generate more animation information [3].

Animation is a kind of digital learning resource, it is an important means to spread information content, and it is also an important online learning resource, including text, image, audio, video, interaction, dynamic effect, their powerful interactive ability in the field of distance education, excellent course website and simulation platform, wide use of this animation and multimedia performance, and accumulated network animation resources [4]. The dynamic learning system is a system that contains many system parameters, including the number of basic decision trees for random forest models and the setting of limit values in the analysis. It is a dynamic learning system [5]. With the necessity of data management of these parameters and the validity time of testing, a part of the dynamic animation learning system is currently semiautomatic, needs system administrators to participate in updating the animation model, ensures the stability and control of the system in the early stages of operation, and gradually reduces the participation manual as the active learning system matures [6]. Learning animation system adopts an active learning method to evaluate some user-driven information. At present, active learning animation system and user interaction mode, from e-mail to user, access automatic animation generation system, and the system administrator evaluates the user in the demonstration database of the animation learning system and studies the animation design application by machine learning and dynamic image index technology.

## 2. Related Work

Some research suggested designing and improving the learning ability of active animation learning system and designing a random forest model for automatic animation production so as to draw lessons from the accumulated animation data and guide animation production [7]. The content structure characteristics of online animation learning resources are comprehensively analyzed, the feature description model of content structure is developed, the description of animation content structure is improved, and the infrastructure of animation content structure is established [8]. The characteristic content of image structure is extracted from a theoretical basis. The animation image structure description model is built to combine color density with edge density to determine the boundaries of the visual scene. Using label data, logical images are extracted from learning resources [9]. The emphasis is on obtaining representative tables through the average master chromatography of each visual scene, the number of which is determined by the number and length of the scene. Based on animation creation principles and related animation techniques, static visual features, visual dynamic effects, and animation interactive processing genes are introduced and quantified through appropriate algorithms [10]. The literature recommends the inclusion of attribute values in the content structure attribute database in order to subsequently identify higher emotional semantics [11]. Based on the content, the literature animated flash semantics representative models, the quantification of abstract emotional semantics into space based on relevant model recognition theories and models, emotional computing, and emotional psychology, combined with the extraction of visual feature vectors using neural network BP, SVM, and the comparative analysis of neural analytic networks, such as learning low-level visual (static visual features and dynamic effects) expressive high-level semantics [12]. To realize the perceptual recognition of images, the literature is explained, mainly by establishing an image index based on K-Means and making a visual dictionary in classification, establishing an image base index, and studying user feedback algorithm [13]. The index results are improved on the basis of information, and the images received from users are searched quickly and effectively.

In this paper, for the first time, an “active” animation learning system using machine learning and dynamic image retrieval technology is designed and implemented [14]. The animation production system can receive the text after selecting the user's favorite background scene and improve the user satisfaction with the animation product. Animation active learning system is closely related to all links of animation system, and animation production and system influence are closely related to these links.

## 3. Design of Dynamic Target Detection Algorithm Based on Machine Learning

### 3.1. Interframe Difference Method

Differential method is the most commonly used method to detect dynamic targets in image sequences, also known as interframe difference method.

The change is detected in the image sequence of the two tables. The time interval between the adjacent image sequence tables is very small, and the constant position of only the dynamic target is changed. Therefore, when the value changes, it can be regarded as the destination. Finally, the moving area is removed, and a dynamic target is achieved by different size threshold, as shown in formula (1):

(1) $$\begin{array}{c} d_{\left(n-1,n\right)}\left(x,y\right)=\left|f_{n}\left(x,y\right)-f_{n-1}\left(x,y\right)\right|. \end{array}$$

Determine dynamic target areas:

(2) $$\begin{array}{c} b_{\left(n-1,n\right)}\left(x,y\right)=\left\{\begin{array}{cc} 1, & d_{\left(n-1,n\right)}\geq T,\\ 0, & d_{\left(n-1,n\right)}<T. \end{array}\right) \end{array}$$

After subtracting every two adjacent frames, the difference image is obtained:

(3) $$\begin{array}{c} d_{\left(n-1,n\right)}\left(x,y\right)=\left|f_{n}\left(x,y\right)-f_{n-1}\left(x,y\right)\right|,\\ d_{\left(n,n+1\right)}\left(x,y\right)=\left|f_{n+1}\left(x,y\right)-f_{n}\left(x,y\right)\right|. \end{array}$$

Then, the binary image is obtained by threshold judgment:

(4) $$\begin{array}{c} b_{\left(n-1,n\right)}\left(x,y\right)=\left\{\begin{array}{cc} 1, & d_{\left(n-1,n\right)}\geq T_{1},\\ 0, & d_{\left(n-1,n\right)}<T_{1}, \end{array}\right) \end{array}$$

(5) $$\begin{array}{c} b_{\left(n,n+1\right)}\left(x,y\right)=\left\{\begin{array}{cc} 1, & d_{\left(n,n+1\right)}\geq T_{1},\\ 0, & d_{\left(n,n+1\right)}<T_{1}. \end{array}\right) \end{array}$$

The dynamic target image of the intermediate frame is detected by logic and operation of the two difference results:

(6) $$\begin{array}{c} M_{k}^{\prime }\left(x,y\right)=d_{\left(n-1,n\right)}\left(x,y\right)\Pi d_{\left(n,n+1\right)}\left(x,y\right). \end{array}$$

*M*′_*k*_ can be converted to

(7) $$\begin{array}{c} M_{k}\left(x,y\right)=M_{k}^{\prime }\left(x,y\right)⊗d_{\left(n,n+1\right)}\left(x,y\right). \end{array}$$

When the pixel value is 1_*k*_ (*x*, *y*), *M*_*k*_ is a dynamic target, otherwise it will be a background.

The frame difference principle (in Figure 1) is very simple. It uses the images in the above table as the current background model and does not accumulate in the calculation. Therefore, its advantages are real-time, fast, and simple. At the same time, because the interval between two adjacent tables is very short, the change in two consecutive tables is not particularly obvious, and the difference in the image is not sensitive to the change of light in the environment.

Background difference method (in Figure 2), also called the background subtraction method, is to model the background and calculate the current image and background in turn.

(8) $$\begin{array}{c} \Delta_{k\left(x,y\right)}=\left|f\left(x,y,k\right)-b\left(x,y,k-1\right)\right|. \end{array}$$

Detection of moving targets is as follows:

(9) $$\begin{array}{c} R_{k}\left(x,y\right)=\left\{\begin{array}{cc} 1, & \text{Foreground }\Delta_{k\left(x,y\right)}>Th,\\ 0, & \text{Background }\Delta_{k\left(x,y\right)}\leq Th. \end{array}\right) \end{array}$$

Basically different, the VCR (video cassette recorder) is static, and it can detect a complete moving target, but the light is sensitive; therefore, providing a background model adapted to the changing environment is crucial for the effectiveness of the method of changing the environment. A number of general background modeling approaches are currently being studied:

(1) Statistical averaging.
Statistical average method is also called the gray level merging method.
  (10) $$\begin{array}{c} B\left(x,y\right)=\frac{1}{k}\sum_{k=1}^{k}f_{k}\left(x,y\right). \end{array}$$
(2) Single Gaussian background modeling.
The gray scale is represented by a Gaussian distribution as follows:
  (11) $$\begin{array}{c} P\left(f\right)=\frac{1}{{\left(2\pi \right)}^{1/2}c_{t}}\exp\left\{-\frac{{\left(f-\sigma_{t}\right)}^{2}}{2\sigma_{t}{}^{2}}\right\}. \end{array}$$
After the model is established, a confidence interval can be obtained. Formula (13) is used to determine the current pixel points:
  (12) $$\begin{array}{c} f\left(x,y\right)=\left\{\begin{array}{cc} 1, & \text{Foreground }\frac{f-\mu_{t}}{\sigma_{t}}>Th,\\ 0, & \text{Background other.} \end{array}\right) \end{array}$$
After judging whether the pixel is a background point, each gray image in the background image needs to be updated:
  (13) $$\begin{array}{c} \left\{\begin{array}{c} \mu_{t}^{*}=\left(1-\alpha \right)u_{t}+\alpha f\\ \sigma_{t}^{2*}=\left(1-\alpha \right)\sigma_{t}^{2}+\alpha {\left(f-\sigma_{t}\right)}^{2} \end{array}\right). \end{array}$$
*α* is a constant that controls the speed of updating.
(3) Codebook background modeling method.

The codewords for a video frame can be expressed as

(14) $$\begin{array}{c} C_{t}\left(x,y\right)=\left[\begin{array}{c} R_{t}\left(x,y\right),G_{t}\left(x,y\right),B_{t}\left(x,y\right),\\ \sigma_{t}\left(x,y\right),f_{t}\left(x,y\right),\lambda_{t}\left(x,y\right) \end{array}\right]. \end{array}$$

**Condition 1 .**

For a given threshold,

(15) $$\begin{array}{c} \text{Coolordist}\left(k\right)=\left\|I\left(x,y\right)-F_{ck}\left(x,y\right)\right\|,\;k=0,1,\ldots ,K. \end{array}$$

When Coolordist (*k*) < the given threshold, the condition is satisfied.

**Condition 2 .**

Determine *a* of adjustment coefficient according to visual characteristics *μ*:

(16) $$\begin{array}{c} \alpha_{u}=\left\{\begin{array}{cc} 10•\mathrm{lg}\left(\mu \right), & \mu \geq \sqrt{255},\\ 10•\mathrm{lg}\left(\sqrt{255}\right), & \mu <\sqrt{255}. \end{array}\right) \end{array}$$

When the brightness is within the confidence interval, the condition is satisfied.

When the two conditions are satisfied at the same time, the minimum codeword is selected as the current matching codeword. Update replacement:

(17) $$\begin{array}{c} \sigma_{k}^{*}\left(x,y\right)=\frac{\text{PowSum}-\left(\text{SumPow}/f_{k}^{*}\right)}{f_{k}^{*}-1}. \end{array}$$

The update rule of the maximum number of rejected lines in codewords is

(18) $$\begin{array}{c} \lambda_{k}^{*}\left(x,y\right)=\max\left\{\lambda_{k}^{*}\left(x,y\right),\lambda_{t}\left(x,y\right)\right\}. \end{array}$$

When it is judged that it does not belong to the same class, the eigenvector of the point is calculated and added to the codebook.

Deletion of scene vector is as follows:

(19) $$\begin{array}{c} \lambda_{t}\left(x,y\right)\geq \frac{N}{2}. \end{array}$$

The basic principle of detecting dynamic targets by the optical flow method (in Figure 3) is to use gray values of dynamic image series to change time zone and stage.

The background and target motion images are determined and calculated, and the Taylor mode of obtaining the optical flow limit equation is amplified:

(20) $$\begin{array}{c} \frac{\partial f}{\partial t}=\frac{\partial f}{\partial x}u+\frac{\partial f}{\partial x}v. \end{array}$$

Assuming that the optical flow is smooth, the speed change rate is 0. At this point, the optical flow should be satisfied:

(21) $$\begin{array}{c} \min\left\{\varepsilon \left(x,y\right)=\sum_{x}\sum_{y}\left\{{\left(f_{x}u+f_{y}v+f_{t}\right)}^{2}\right\}\right\}. \end{array}$$

The optical flow estimation error is defined as

(22) $$\begin{array}{c} \varepsilon =\sum_{\left(x,y\right)\in \Omega }W^{2}\left(x\right){\left(f_{x}u+f_{y}u+f_{t}\right)}^{2}. \end{array}$$

Among them, *W*^2^(*x*) represents a window weight function. Among the LK algorithms, some cases will lead to the irreversibility of the matrix, and the design error is very large when the object has a large range of motion.

### 3.2. Classic Machine Learning Algorithm

BP neural network model is a three-layer structure, including input layer, hidden layer, and output layer. When input data *Xn* is from the first input layer to the second hidden layer, the following mathematical model shall be converted:-

(23) $$\begin{array}{c} Q_{1}=f\left(P_{11}x_{1}+P_{12}x_{2}+P_{13}x_{3}\ldots +P_{1n}x_{n}+b_{1}\right)\\ Q_{2}=f\left(P_{21}x_{1}+P_{22}x_{2}+P_{23}x_{3}\ldots +P_{2n}x_{n}+b_{2}\right)\\ Q_{3}=f\left(P_{31}x_{1}+P_{32}x_{2}+P_{33}x_{3}\ldots +P_{3n}x_{n}+b_{3}\right)\\ \cdots \\ Q_{n}=f\left(P_{n1}x_{1}+P_{n2}x_{2}+P_{n3}x_{3}\ldots +P_{nn}x_{n}+b_{n}\right). \end{array}$$

Among them, *P*_*ij*_, which is the weight between layers, is an important parameter affecting the accuracy of the model, from the second hidden layer to the third layer.

The following mathematical models should be transformed:

(24) $$\begin{array}{c} y_{1}=Q_{1}=f\left(P_{11}x_{1}+P_{12}x_{2}+P_{13}x_{3}+\cdots +P_{1n}x_{n}+b_{1}\right)\\ y_{2}=Q_{2}=f\left(P_{21}x_{1}+P_{22}x_{2}+P_{23}x_{3}+\cdots +P_{2n}x_{n}+b_{2}\right)\\ y_{3}=Q_{3}=f\left(P_{31}x_{1}+P_{32}x_{2}+P_{33}x_{3}+\cdots +P_{3n}x_{n}+b_{3}\right)\\ \cdots \\ y_{4}=Q_{n}=f\left(P_{n1}x_{1}+P_{n2}x_{2}+P_{n3}x_{3}+\cdots +P_{nn}x_{n}+b_{n}\right). \end{array}$$

### 3.3. Improved Foreground Target Extraction for Five-Frame Difference by Fusion

Save the same information to the maximum extent, and dynamic targets such as background pixels are accurately preserved, but this also means that there will be more targets. The image operations *N*_1_ (*X*, *Y*) and *N*_2_ (*X*, *Y*) ensure the removal of the moving target area. *N* of results_1_ (*X*, *Y*) *N* results_2_ (*X*, *Y*) Postaction *M* to outcome_1_*X*, *Y* and *M* of results_2_ (*X*, *Y*) “Same or”

Conduct “transactions” to obtain

(25) $$\begin{array}{c} s_{1}\left(x,y\right)=m_{1}\left(x,y\right)⊗n_{1}\left(x,y\right)=\left\{\begin{array}{cc} 1, & m_{1}\left(x,y\right)\Pi n_{1}\left(x,y\right)=1,\\ 0, & m_{1}\left(x,y\right)\Pi n_{1}\left(x,y\right)\neq 1, \end{array}\right) \end{array}$$

(26) $$\begin{array}{c} s_{2}\left(x,y\right)=m_{2}\left(x,y\right)⊗n_{2}\left(x,y\right)=\left\{\begin{array}{cc} 1, & m_{2}\left(x,y\right)\Pi n_{2}\left(x,y\right)=1,\\ 0, & m_{2}\left(x,y\right)\Pi n_{2}\left(x,y\right)\neq 1, \end{array}\right) \end{array}$$

where *s*_1_(*x*, *y*) and *s*_2_(*x*, *y*) perform “or” operations to obtain the final target area *m* (*x*, *y*); namely,

(27) $$\begin{array}{c} m\left(x,y\right)=s_{2}\left(x,y\right)\cap s_{2}\left(x,y\right)=\left\{\begin{array}{cc} 1, & m_{2}\left(x,y\right)∐n_{2}\left(x,y\right)=1,\\ 0, & m_{2}\left(x,y\right)∐n_{2}\left(x,y\right)\neq 1. \end{array}\right) \end{array}$$

The maximum interclass variance method is used to set the binarization threshold, which further improves the extraction speed, and the illumination information is also integrated into the threshold judgment:

(28) $$\begin{array}{c} \max\left|\Delta h_{k}\left(x,y\right)\right|>T+\gamma \frac{1}{N}•\sum \left|\Delta h_{k}\left(x,y\right)\right|. \end{array}$$

Gamma value is the premise that the basic light does not change. When the light changes, the gamma value rises, and the judgment threshold rises, thus reducing light to a certain extent. These changes reduce the effect of light on the accuracy of test results.

### 3.4. Comparative Analysis of Experimental Results

The research on the above three kinds of target dynamic detection algorithms shows that each kind of target is in a specific environment. As shown in Table 1, the three algorithms in the current table should be more clearly explained for each of the three algorithms applying different environmental conditions.

In order to show the effect of the algorithm test more intuitively, two videos have been taken, the real animation of the same image has been taken, and the image contrast analysis is carried out directly on the interface. The difference between the two tables is most obvious in the internal extraction of dynamic targets. Animation and coverage are not allowed to extract target graphics and are not very effective. Three different tabular methods also allow to appear on the screen in the form of clear and nonrepeated borders, extracting graphics from dynamic targets, but with some flaws in the targets. Under variable light conditions, the overall defect of the measurement target cannot be extracted from the target and cannot be rehearsed. GMM animation can get the outline of the target animation icon, but it is affected by light; there will be some shortcomings, and the animation algorithm running speed is shown in Table 2.

In principle, for a good dynamic target detection algorithm, the following conditions should be satisfied:

1. Insensitive to slow changes in the environment.
2. Can handle complex background and complex target situation.
3. Can adapt to the interference in the environment.
4. Can reduce the shadow effect of the algorithm results.
5. Meet the accuracy requirements of subsequent processing such as identification.

The above dynamic target testing algorithm meets the requirements of accuracy and can be processed for a long time, and the operation time is very short. The algorithm cannot detect the whole target; everyone has a real disadvantage. ADEM in these algorithms: many can be used, and each algorithm of different applications can be used in different applications. *K*-Means clustering algorithm can process a large number of high-resolution impact data sets; these data sets are simple and effective and have been applied. Nevertheless, the average *K* itself has many defects, the first of which is the *K* value, which is determined in some complex environments. It should be a dynamic value for change, and sometimes manual estimation of experience and applied data sources in the PRA is required. Several attributes of the main data set are selected as cluster centers. However, if the difference between the data sets is not very clear and the density of the data sets has many noise points, the results of the data sets are often not very stable or effective. Given the initial group concentration, the algorithm is selected to minimize the value of the objective function. However, when the selection value is not appropriate, the result is often the best result locally, and the understanding of the destination function is not as good as possible. Image attributes should be minimized to speed up the retrieval and optimization of random starting points of the K-means group algorithm. In order to improve the application of visual dynamic image search help, animation designers can understand the current popular animation style and content and better design and production of animation.

In order to ensure that the results of the enhanced algorithm combination are better than those of the randomly determined initial central cluster, the distance between the classification centers should be judged according to the degree of separation of the classification. The difference between the grouped data and the central values of the aggregate level in the classification is used to judge. When calculating the higher value of the grouping result, the greater the distance between the classifications, the higher the level and the longer the edge description algorithm works for all levels.

First, as shown in Table 3, the interval distance between K-Means classification results is larger than that between K-Means normal classification results, and its interval distance is less than that of K-Means. This indicates that if SITF point coordinates are used to group in different image groups, the effect of the enhancement algorithm group is the greatest. ADEM is the improvement of the K-Means cluster, which requires less repetition times and is more effective. The K-Means algorithm is shown in Table 4.

## 4. Application of Machine Learning and Dynamic Image Index in Animation Design Generation

With the development of the times, information technology and our life are closely linked, and information technology affects all levels of our daily life; every angle of our daily life cannot be separated from information technology. Education is very important for the development of a country. Education embodies the future of a nation. The combination of education and information technology can open up a new development path for educational practice and accord with the development trend of the new era. With the development of the times, animation plays an increasingly important role in our daily life. It is no longer the exclusive film to educate children; animation can be closely linked with people's daily life through information technology for the development of the animation industry into a new development power. At present, the development of information technology promotes the development of artificial intelligence technology, and artificial intelligence technology is very popular in today's era. It is a machine learning chip. Artificial intelligence technology can combine animation creation, identify, classify, and process some animation data, organize some animation works, and search the images of animation works. In the past, the scope of image retrieval was very small, limited to the three aspects of article content, semantics, and text. With the popularization of artificial intelligence technology, the scope of image retrieval technology is gradually expanding. People can fully use machine learning to retrieve content but also add artificial intelligence recognition and data recognition and further improve the accuracy of image retrieval. Image retrieval and animation design can also be combined to improve the animation creation efficiency of creators.

### 4.1. Automatic Animation Generation Based on Machine Learning

The automatic animation production system is based on artificial intelligence technology, receives the text information after natural processing and semantic analysis, then takes the text as the starting point, carries on the qualitative and quantitative analysis of the animation environment, and finally carries on the production.

Acoustic animation and synthesis for output animation. The procedures are shown in Figure 4.

As a whole, the automatic animation production system has successfully adopted a knowledge-based method. Therefore, this paper develops a dynamic animation learning system for automatic animation production system using a random forest model. Learn from a large amount of accumulated information, this information can guide animation production through the animation production system, and actively learn how to let users participate. Users and managers interact to achieve learning. The learning machine is divided into supervised learning and semisupervised active learning. As a means of semisupervised learning, it is a progressive sample prediction method. It can select some unlabeled samples according to some principles, actively communicate with the outside world to obtain the true marks of these samples, and then use these samples to complete the research marks. Compared with the general semimonitoring learning method, active learning can greatly reduce the demand for samples through similar correction rates, and the active learning process can be shown in Figure 5. Experimental determination of optimal relative parameters of random forest model and comparative experiment of decision tree model show that random forest model automatically produces advantages through animation. At the same time, two sets of experiments are designed to verify the feasibility and effectiveness of the active animation learning system.

The active learning animation system is based on the experimental results and uses the random forest model as the learning model, which includes 11 decision trees with an error rate of 0.21. In order to solve these two problems, we have been expanding, on the one hand, with the operation of animation production system; on the other hand, the parameters of the random forest algorithm are adjusted through new experiments.

Active learning animation system uses the historical data of user animation product evaluation and animation system as training samples and uses the machine learning algorithm to produce a classification model based on user evaluation in order to guide the animation production system, to produce the most satisfactory animation. However, the user's evaluation of animation is a subjective judgment; The user's understanding of the text, the user's psychological state, color, music, and the movement of the animation itself will affect the evaluation results. Therefore, an active learning system is needed to help the animation production system select a preferred background scene. The decision tree model is used to improve the satisfaction of animation product users and reduce the error rate.

### 4.2. Animation Design Based on Dynamic Image Retrieval

The overall features of an image are general image information, in which the most common features are color, texture, and graphics. Some search systems use the features of images to build image search indices because the advantages of these features include variability, simple computation, and visualization. Search of image index is shown in Figure 6.

Because of the benefits of related search, it is inevitable to apply it to image retrieval, especially in the aspect of the “semantic gap” in image-based image retrieval. This is mainly because the user's abstract interpretation of the image, the use of visual descriptions such as background color, shape in the CBIR, and the differences between high-level semantics and background visual features may lead to unsatisfactory search results. Therefore, the content-based image retrieval feedback process requires continuous capture of images. After multiple interactions between the user and the system, the user needs to fully incorporate the user's subjective views into the system.

## 5. Realization of Animation Design Based on Machine Learning and Dynamic Image Indexing Technology

### 5.1. Completion of Animation Design

The active animation learning system designed in this paper allows the continuous receiving of sample data from the animation system and the automatic expansion of the sample number through interaction with the animation production system, users, and managers to carry out the “initiative action.” The algorithm is used for active learning, selecting samples that need to interact with users, and solving problems. Because the KFF method does not take into account the diversity of samples to be marked, the active animation learning system uses statistical methods to learn the uniqueness of samples.

3D animation automatic production system faces two challenges: (1) there may be a lack of learning ability and waste of a large amount of animation information data accumulated since the system was launched in 2008; (2) the quality of animation produced depends on the level of system designers. Users of the system cannot participate in the production of the system. It was originally designed for animation production system and implemented a dynamic animation learning system so that the animation production system can continue to learn experience and produce the most popular animation users.

### 5.2. Learning Ability of Active Animation Learning System

First, the master designed a random forest model for automatic animation production to draw lessons from accumulated animation data, guide animation production, implement animation production systems, and abstractly develop the characteristics and categories of random forest models; standardize large amounts of historical data and receive training samples for random forest model development; and continuously test and optimize random forest model parameters so that the learning model can better guide animation production systems to form a complete system user: active learning animation system, “active” learning ability developed.

Secondly, the animation active learning system designed in this paper interacts with the animation production system, system users, and managers so that the sample data of the system can be continuously received, the number of training samples is automatically expanded, the status of the sample database is analyzed, and suggestions for updating the learning model are made to the system managers when necessary. We use KFF algorithms and K-Means statistics to actively learn and select samples that need to interact with users.

Through the subjective interpretation of the image, the image content is summed up into the key text, time, place, and image text information to determine the correlation of the image and ensure that the image becomes text. This method is relatively simple, but with the increase of image volume, the labor consumption of manual text identification is also increasing, the subjectivity of manual identification is also increasing, and the content of text summary image is not comprehensive. This may lead to differences in image understanding and defects in text description.

### 5.3. Shortcomings in Animation Design

At the same time, a number of experiments in active learning animation systems have identified potential problems and deficiencies requiring further research, including the following.

First, expand model learning. The animation active learning system designed in this paper is based on the choice of background animation scene. It is necessary to further study whether this learning model based on background scene can be extended to the model.

Secondly, optimize the parameters of dynamic animation learning system. Dynamic learning system is a system that contains many parameters of the system, including the number of basic decision trees of random forest models. Limit configuration in data management analysis, the necessity of further testing these parameters, and the validity of time testing.

Third, reduce the participation of system users and managers. The dynamic animation learning system is semiautomatic and needs system administrators to participate in updating the animation model. Manual participation ensures that, in the initial stage of system operation, the stability and control of the system and the maturity of the active learning animation system will need to gradually reduce the participation of manual operation. On the other hand, the active animation learning system adopts a positive learning method to obtain the user's evaluation of part of the animation text. Now, the active animation learning system interacts with the user by displaying the amount of text information. Users can use the 3D animation automatic generation system generated by automatic animation to find digital short messages that need assessment. System administrators evaluate users of the sample database of active animation learning system. In the next version of the active animation learning system, a more direct and faster interface can be established for users.

Based on the advantages of animation, students need to regain the learning resources of online animation. This study has begun to analyze and restore the structural features of the content of online learning resources. By analyzing the content of animation learning resource files, visual scenes and their visual features extraction, composition elements characteristics, internal animation graphics, emotional features, and so on, a database with animation content structure characteristics will be created, which will eventually be used in a network-based dynamic learning resource search system. This study is very important in theory for the educational application of learning animation resources on the Internet and confirms that animation content has a positive impact on students' interest in learning. It complements the model of applying online animation resources in teaching and enriches the content of online learning resources. The analysis of content structure features helps to improve the efficiency of finding learning resources. Animation is based on rich dynamic image content to introduce knowledge to students. In many cases, students express emotional content according to the characteristics of animation content, such as tone, texture, dynamic effect, and button. Through the content-based Internet developed by the Institute, the animation search system can improve the efficiency and accuracy of searching for learning resources on the Internet and increase the use of Internet animation resources. It strengthens the self-study contribution of many students and provides educational information services.

## 6. Conclusion

Information technology has been integrated into all aspects of work, life, and learning. Adopting the development concept of “Educational Informatization 2.0”, information technology and educational practice are deeply brought into the development trend, and animation is becoming more and more important in our life. It is very important to explore the role of new technology in animation design. Machine learning is the basic technology of artificial intelligence at present, which can be very helpful to determine the characteristics of animation. The research experience of image retrieval technology is based on three stages: text, content, and semantic search. These stages mainly rely on semantic image search, including machine learning knowledge, content retrieval-based artificial intelligence, model recognition, and data extraction, in order to improve resilience genes. Animation is also an important medium for transmitting information today. It not only is an entertainment media but also carries the function of learning. Animation is a kind of multimedia interactive ability and expressive ability. Animation is used not only in entertainment but also in teaching. In order to establish an animation active learning system, the animation resources can be summarized, the automation state of the animation learning system can be improved, the stability of the animation learning system can be guaranteed, and the animation active learning system can be matured as soon as possible. The application of image retrieval to the design and production of animation enables producers to understand the current trend of animation production. The role of these two techniques in animation image design enables animated images to better adapt to people's aesthetics and guide the future.

## Figures and Tables

**Figure 1:** Frame difference method.

**Figure 2:** Background difference method.

**Figure 3:** Schematic illustration of the pyramid optical flow method.

**Figure 4:** Schematic diagram of interactive content.

**Figure 5:** Flowchart of active learning.

**Figure 6:** Establishment and search of image index.

**Table 1:** Comparison of three dynamic target detection methods.

	Interframe difference method	Background difference method	Optical flow method
Operation complexity	Small	Middle East	Large
Operation speed	Hurry	Slow	Slow
Scope of use	Background relatively fixed	Background relatively fixed	Background removable
Results of operations	The entire region of the dynamic target cannot be extracted, and the contour is incoherent	The whole area of the dynamic target can be obtained, and time-consuming modeling is sensitive to light	The dynamic effect can be obtained in the whole area, but it is easy to be affected by noise and difficult to apply

**Table 2:** Comparison of four algorithms.

	2-frame difference method (fps)	3-frame difference method (fps)	SGM (fps)	GMM (fps)
Highway	1	1	12	8
People	2	3	36	32

**Table 3:** Cluster results.

Algorithm	Average distance between classes	Average variance within class	Number of iterations	Duration (ms)
K-Means algorithm	277.252	36.672	23	1643
An improved K-Means algorithm	344.887	22.954	11	560

**Table 4:** Improved K-Means algorithm.

Input	User input data set *s* for clustering and *T* maximum number of iterations
Output	Clustering of *K* clusters.

1	Scan the original data set to find the two data points with the largest distance as the initial clustering center C, and the *K* is 2.
2	Referring to the maximum and minimum clustering method, the distance from each point to each cluster center in the data set is viewed, and the shortest distance is taken and recorded.
3	The shortest distance from each point to each type of center is compared, and the data point with the maximum distance is taken as the candidate of the new cluster center. At this time, the previous cluster center should be saved to find that the cluster center candidate is not suitable and goes back to the previous result. The result of the new cluster center should be reclustered, the cluster center should be updated, and the value DBI the objective function should be updated for the K+ cluster.
4	According to the previous analysis, it is judged whether the new *K* value can be the result of clustering to reach the optimal solution. As the DBI calculation results become smaller than the last time, it is proved that the new cluster center point is better; we should go back to the second step and continue to iterate. If the result is larger than the last time, the last *K* value should be optimal; return to the last cluster center, and jump to step 5.
5	The result of the optimal *K* is obtained, and the clustering result satisfies the optimal solution of the objective function and returns *K* cluster result clusters.

## Data Availability

The data used to support the findings of this study are currently under embargo while the research findings are commercialized. Requests for data, 6 months after publication of this article, will be considered by the corresponding author.
